# Polyacetylenes from *Codonopsis lanceolata* Root Induced Apoptosis of Human Lung Adenocarcinoma Cells and Improved Lung Dysbiosis

**DOI:** 10.1155/2022/7713355

**Published:** 2022-02-18

**Authors:** Meng-Chuan Wang, Yu-Fang Wu, Wen-Ying Yu, Bing Yu, Hua-Zhong Ying

**Affiliations:** ^1^Zhejiang Key Laboratory of Experimental Animal and Safety Evaluation, Zhejiang Academy of Medical Sciences (Hangzhou Medical College), Hangzhou 310013, China; ^2^College of Pharmaceutical Science, Zhejiang Chinese Medical University, Hangzhou 310053, China

## Abstract

*Codonopsis lanceolata* is a perennial smelly herbaceous plant and widely employed for the treatment of various lung cancer and inflammation. However, the anticancer substances in *C. lanceolata* and their underlying mechanisms had not been well clarified. In this study, six compounds were obtained from the water extracts of *C. lanceolata* polyacetylenes (CLP) and then identified as syringin, codonopilodiynoside A, lobetyol, isolariciresinol, lobetyolin, and atractylenolide III. Treatment with CLP remarkably suppressed the cell proliferation, colony formation, migration, and invasion of A549 cells. Synergistic effects of lobetyolin and lobetyol were equivalent to the antiproliferative activities of CLP, while other compounds did not have any inhibition on the viabilities of A549 cells. CLP also reduced the expression of Ras, PI3K, p-AKT, Bcl-2, cyclin D1, and CDK4 but increased the expression of Bax, GSK-3*β*, clv-caspase-3, and clv-caspase-9, which could be reversed by the PI3K activator 740YP. Furthermore, CLP retarded the growths of tumor and lung pathogenic bacteria in mice. It demonstrated that lobetyolin and lobetyol were the main antitumor compounds in *C. lanceolata*. CLP induced cell apoptosis of lung cancer cells via inactivation of the Ras/PI3K/AKT pathway and ameliorated lung dysbiosis, suggesting the therapeutic potentials for treating human lung cancer.

## 1. Introduction

Lung cancer is presently one of the most harmful human diseases with the highest morbidity throughout the world, which has an incidence of 20.9 million new cases and 18.0 million deaths in 2018 [1]. The occurrence and development of lung cancer involve various complex pathological mechanisms and are prone to metastasis to the bone, brain, liver, and lymph node, resulting in the trick reversion in clinic [2–4]. Although chemotherapy has been a major means for lung cancer therapy, prolonged, repeated intravenous chemotherapy causes drug resistance and several side effects [5, 6].

In recent years, traditional Chinese medicines have played a prominent part in tumor growth, immune function, and life expectancy for the treatment of lung cancer [7, 8]. *Codonopsis lanceolata* (family *Campanulaceae*) is a dicotyledonous herbaceous perennial plant mainly distributed in the northern parts of China, Russian, and North Korea. The roots of *C. lanceolata* are used as a folk medicine for treating various lung diseases, including cough, bronchitis, edema, asthma, and lung cancer over thousands of years [9–12]. It contains a wide variety of distinctive metabolites (e.g., polysaccharides, saponins, and polyacetylenes) [9, 13, 14]. It has been reported that the n-butanol extract of *C. lanceolata* root induced the apoptosis of human colon cancer HT-29 cells via ROS accumulation and polyamine depletion [15]. Its methanol extract also induced the apoptosis of human oral cancer HSC-2 cells through activation of the Bak pathway [16]. Codonoposide 1c, an echinocystic acid derivative obtained from the root of *C. lanceolate*, triggered caspases-dependent apoptosis in acute myeloid leukemia HL-60 cells [17]. In addition, the water extract of *C. lanceolata* attenuated various stimuli-induced lung inflammation by inhibiting alveolar macrophage and Th2 cell activation, indicating its anti-inflammatory potential on respiratory inflammatory diseases [12, 18, 19]. However, previous studies mainly focused on the quality control and structure analysis of various chemical components from *C. lanceolata*. The ingredients responsible for the anticancer effects of *C. lanceolata* and their underlying mechanisms remain unknown. In the present study, the polyacetylenes of *C. lanceolata* (CLP) loaded onto the chromatographic column to the bioactive polyacetylenes of *C. lanceolata* (CLP) were yielded through silica gel chromatography separation, and then, their antitumor potentials were assessed in A549 cells and in tumor-bearing mice.

## 2. Materials and Methods

### 2.1. Materials and Reagents

Fetal bovine serum (FBS) was acquired from Tianhang Biotech. Co. Ltd., Hangzhou, China. MTT was obtained from Sigma-Aldrich (China). Antibodies used in the study were obtained from Cell Signaling Technology (Danvers, USA) or Abcam (Cambridge, UK). Other regents were all purchased from Hangzhou Bozan Biotech. Co. Ltd., China.

### 2.2. Extraction and Isolation of Compounds in CLP

The isolation process was based on the related articles with minor changes [20–22]. The herb was purchased from the Zhejiang Traditional Chinese medicine factory, appraised by Dr. Xiong-Ning Wu in our college, and the rest of the samples were stored in a specimen room (no. 2019W0512). The air-dried plants (20 kg) were extracted 2 times (boiling 1 h with 200 L of water each time). The water extract was concentrated to be 30 kg of weight and then mixed with 45 L of 95% ethanol overnight. The supernatant was concentrated and then purified by AB-8 macroreticular resin. After being eluted with 80% alcohol, the eluent was collected and then dried by hypobaric drying to yield the purified extract (CLP, 2.6 kg). This extract CLP was subsequently subjected to column chromatography over HP-20 resin (100–200 mesh) and separated with a gradient elution [H_2_O–EtOH (4 : 1–1 : 1, *v*/*v*)]. Compounds 1 (10.2 mg), 2 (8.8 mg), 3 (10.6 mg), 4 (20.5 mg), 5 (94.3 mg), and 6 (37.9 mg) were found from 50% EtOH− elution by the preparative HPLC system. The purities of these compounds were analyzed by using HPLC.

### 2.3. Quality Control of CLP

The CLP or each isolated compound was prepared by dissolving in methanol. After filtering through a 0.22 *μ*m membrane, 20 *μ*L of the sample was subjected to the HPLC system. The HPLC column was a Kromasil C_18_ column (250 mm × 4.6 mm, 5 *μ*m). The temperature was kept at 30°C during the whole analytical process. The detection wavelength was 220 nm. The flow rate of the mobile phase (acetonitrile (A) and 0.1% phosphoric acid (B)) was 1.0 mL/min. The conditions of elution were set as follows: 0–20 min, 10% A; 20–30 min, 10% A⟶30% A; 30–40 min, and 30% A⟶70% A. The resolution of each compound was not less than 1.5. The theoretical plate numbers of syringin should be larger than 5000.

### 2.4. Cell Viability and Colony Formation Assays

The cells were seeded into the 96-well plates (each well had 5000 cells) and then treated with CLP (2.5, 5, and 10 *μ*g/mL) or DDP (5 *μ*g/mL) for 24, 48, and 72 h. Twenty microliters of PBS solution containing 5 mg/mL of MTT was assigned to each well and incubated at 37°C for 4 h. At last, each well was mixed with 150 *μ*L of dimethyl sulfoxide. The absorbance was measured at 490 nm.

Cells were seeded into six-well plates (10^3^ cells/well) and then treated with CLP (2.5, 5, and 10 *μ*g/mL) or DDP (5 *μ*g/mL). When a clearly visible colony appeared in the culture dish, the cells were fixated with methanol and subsequently dyed with 10% Giemsa for 10–30 min. Colonies were counted under an optical microscope (OLYMPUS, Japan).

### 2.5. Transwell Invasion and Wound Healing Assays

The serum-free medium containing 1 × 10^5^ cells were added into the upper chambers of the transwell chambers (8 *μ*m pore size) with Matrigel (BD Biosciences, USA), while 500 *μ*L of 20% FBS medium was presented into the matched lower chambers. Forty-eight hours after incubation with test drugs, only the lower chambers were collected, fixated with methanol for 30 min, and stained with 0.1% crystal violet for 15–30 min. The cells on the lower surfaces of the chambers were counted under the optical microscope (OLYMPUS, Japan).

The cells were seeded into six-well plates (each well had 2.5 × 10^5^ cells). The cell layer of each well was wounded by using the tip of a 200 *μ*L pipette. The wells were carefully washed with PBS to remove the detached cells, and then, the remaining cells were cultured at 37°C for 48 h. Images were captured at 0 and 48 h after scratching, and the wound width in each well was measured with a ruler under the microscope (OLYMPUS, Japan).

### 2.6. Cell Apoptosis and Cell Cycle Assay

The cells in 6-well plates were treated with CLP at the concentrations of 2.5–10 *μ*g/mL for 24 h and then mixed with 500 *μ*L of buffer, 5 *μ*L of annexin V FITC (20 *μ*g/mL), and 10 *μ*L of PI (50 *μ*g/mL). The apoptotic rates of CLP-treated A549 cells were detected by using flow cytometry (BD, USA). On the other hand, the cells were also collected for examining cell cycle distribution according to the commercial kit (MultiSciences Biotech Co. Ltd., Hangzhou, China). Cells were treated with 500 *μ*L of buffer and 5 *μ*L of permeabilization solution and then kept for 20 min at room temperature and no-light conditions. Finally, the cell cycles of stained cells were assayed by flow cytometry.

### 2.7. Western Blot Assay

The total proteins of cells or tumor samples were extracted with 0.2 mL of RIPA, 1 *μ*L of PMSF, and 1 *μ*L of the phosphorylation protease inhibitor. Then, the supernatant of the protein extracts was collected and its quality was controlled by the BCA detection kits (KeyGEN BioTECH Co. Ltd., Nanjing, China). The total proteins were diffused on 12% SDS-PAGE electrophoresis and transferred onto the polyvinylidene difluoride membranes. These membranes were soaked in 5% nonfat milk for 2 h and then treated with primary antibodies for 10 h at 4°C. After pretreatment with TBST for 3 times, the membranes were treated with secondary antibodies for 1 h. The expression of the target proteins was measured by using chemiluminescence (Beyotime, China). GAPDH was considered as the control for Western blot analysis.

### 2.8. Animals and Experimental Procedure

Thirty male nude mice (six weeks old) were provided from Shanghai SLAC Co. Ltd., China. Those mice were fed in the specific pathogen-free conditions (room temperature, 22–24°C; humidity, 45–55%). The operational process followed the guidelines of our college and was approved by the ethics committee of the college (no. 2020R0505).

Approximately 5.0 × 10^5^ cells of luciferase-overexpressing A549 cells were injected into the left lung of each nude mouse to prepare a xenograft mouse model as recent reports [23–25]. The tumor-bearing mice after one-week postinjection were randomly divided into the five groups: (1) model group, intragastrical administration (i.g.) with 10 mg/kg of saline; (2) CLP-L group, i.g. 10 mg/kg of CLP; (3) CLP-M group, i.g. 20 mg/kg of CLP; (4) CLP-H group, i.g. 40 mg/kg of CLP; and (5) DDP group, i.g. 5 mg/kg of DPP. Each group had six mice. The mice in the model and CLP groups received oral administration once a day for 15 days, while the mice in DDP-treated group were intraperitoneally injected once every 3 days. The weighs of mice were recorded every 3 days.

The growth of orthotopic tumor was monitored every 5 days by using the IVIS Lumina LT imaging system (PerkinElmer, USA). Briefly, the mice were anesthetized by isoflurane and then intravenously injected with 1.5 mg D-luciferin (Yeasen, China) 10 min prior to imaging.

### 2.9. HE and TUNEL Assays

Tumor tissues were soaked in 4% formaldehyde for more than 96 h, and then, the cured samples were pretreated with gradient ethanol and finally put into the paraffin. Tumor samples were stained by hematoxylin and eosin (HE) solution. Furthermore, the apoptotic cells in tumor tissues were marked by using an in situ apoptosis detection kit (Roche, USA). The images of positive cells (presented green fluorescence) were captured under fluorescence microscopy (Zeiss, Germany).

### 2.10. Immunohistochemistry

Tumor tissues were prepared as in Section 2.9. The paraffin-embedded samples excised from A549 nude mice were stained by using Ki-67 and pAKT antibodies for immunohistochemistry. Images of the tumor tissues were captured using a light microscope (Leica DM2500, Germany).

### 2.11. Bacterial 16S rDNA Sequencing

The bacterial diversity and abundance of lung samples were analyzed by 16S rDNA sequence analysis [26, 27]. The total DNA was extracted using DNA extraction kit (Tiange, China). The DNA quality and purity were controlled by using the NanoDrop ND-1000 system (Thermo, USA). The 16S rDNA genes of the V3-V4 regions were amplified by using a specific primer (F:5′-ACTCCTACCGAGCAGAGAG-3′, R:5′-GGACTACHgGT WTCTATT-3′) with the barcode. The reaction parameters were set as initial denaturation at 98°C for 30 s, followed by 32 cycles of denaturation at 98°C for 10 s, 54°C for 30 s, and 72°C for 45 s and annealing at 72°C for 10 min. Agilent 2100 Bioanalyzer (Agilent, USA) was used to prepare and evaluate the library, and Illumina's library quantification kit (Kapa Biosystems, USA) was used for quantification. The amplified library was sequenced on Illumina NovaSeq PE250 platform according to the standard steps (2 × 250) by LC Biotech. Co. Ltd. (China).

### 2.12. Detection of Antibacterial Activity of CLP

*Streptococcus pyogenes* (CVCC1882) and *Staphylococcus aureus* (CVCC376) were donated by Dr. Fanwei Dai, Zhejiang Animal Research Center, China. The minimum inhibitory concentration (MIC) and the minimum bactericidal concentration (MBC) of CLP on these two tested strains were measured in vitro by the 2-time dilution method and decided visually according to the presence or absence of strains [28–30]. Each concentration was detected 5 times. The plates were cultured at 37°C for 24 h. To detect MBC values, the concentrations of CLP tested in the study were higher than its MIC values. Moreover, the filter paper was made into a circular paper with a diameter of 5 mm and sterilized for further use. The filter papers with the prepared test solution were placed on the solid media and applied evenly with bacteria solution. The diameters of the inhibition zone of samples were determined 24 h after treatment.

### 2.13. Statistical Analysis

Each assay was performed 3 times. The data were showed as the mean ± standard deviation (SD). Statistical differences were analyzed by one-way ANOVA by using the GraphPad Prism 6 and SPSS 16.0 software. The significant differences between 2 groups were set at *P* < 0.05.

## 3. Results

### 3.1. Chemical Analysis of Compounds in CLP

Six compounds were isolated from *C. lanceolata*, and their structures were characterized as syringin (1), codonopilodiynoside A (2), lobetyol (3), (+)-isolariciresinol (4), lobetyolin (5), and atractylenolide III (6) by comparing their physical and spectral data (HR-MS, HPLC, ^1^H-NMR, and ^13^C-NMR) with previous reports [20–22, 31, 32]. Among those compounds, compounds 2, 4, and 6 were first found in the plant *C. lanceolata*.

To control the quality of the herbal extract CLP, we determined the contents of the six compounds by HPLC. The representative HPLC chromatograph was presented as shown in Figure 1(a). The contents of syringin, codonopilodiynoside A, lobetyol, (+)-isolariciresinol, lobetyolin, and atractylenolide III in CLP were 46.9%, 5.7%, 9.3%, 12.6%, 10.5%, and 1.1%, respectively.

### 3.2. Effect of CLP on A549 Cell Proliferation

The results in Figure 1(b) showed that CLP remarkably inhibited the proliferation of A549 cells in time- and concentration-dependent manners 24–72 h after administration with 1.25–20 *μ*g/mL of CLP, respectively. The IC_50_ values of CLP on A549 cell proliferation for 24, 48, and 72 h were 13.5, 10.5, and 8.6 *μ*g/mL, respectively. Most notably, treatment with 20 *μ*g/mL of CLP for 24–72 h did not affect the viabilities of human normal lung epithelial BEAS-2B cells (Figure 1(c)), suggesting its low cytotoxicity.

To determine the anticancer pharmacodynamic substances in CLP, the six compounds isolated from CLP were investigated *in vitro* in A549 cell model. As shown in Figure 1(d), lobetyol, lobetyolin, and atractylenolide III had significant inhibition on the cell proliferation of A549 cells, while other compounds showed little or no effects. Considering that the contents of those six compounds in CLP were clear, the contribution of each compound to the antiproliferative activities of CLP could be calculated by comparing their overall and individual inhibition. The inhibitory rates of CLP (20 *μ*g/mL), syringin (9.38 *μ*g/mL), lobetyol (1.86 *μ*g/mL), lobetyolin (2.10 *μ*g/mL), and atractylenolide III (0.22 *μ*g/mL) on the proliferation of A549 cells were 65%, 8.1%, 21.8%, 24.4%, and 2.3%, respectively. Therefore, lobetyol and lobetyolin contributed approximately 71% to the inhibitory effects of CLP on lung cancer cell proliferation (Figure 1(e)). Although the content of syringin in CLP was approximately fivefold higher than those of lobetyol and lobetyolin, the antiproliferative activity of syringin was approximately fourfold less. Thus, lobetyol and lobetyolin could be the main anticancer compounds. Moreover, the combination index of lobetyol and lobetyolin, which were mixed at 5 different concentrations (Figure 1(f)), was around the additive baseline 1, indicating their additive effects.

### 3.3. Effects of CLP on A549 Cell Migration, Invasion, and Colony Formation

As shown in Figure 2, the width of wound scratch in the control group was significantly reduced 48 h after CLP treatment. However, compared with the untreated group, wound closures were significantly decreased in the CLP-treated groups (*P* < 0.05), indicating the inhibition of CLP on A549 cell migration. Moreover, the results of transwell assay showed that approximately 250 cells invaded the lower chamber in the control group after CLP treatment for 48 h. However, the number of cells in the lower chamber was significantly decreased in the CLP-treated groups compared with the control group (*P* < 0.05), indicating the inhibition of CLP on A549 cell invasion. Similarly, CLP dose dependently inhibited the colony formation of A549 cells. But colonies were hardly found in 10 *μ*g/mL of the CLP-exposed group.

### 3.4. Effects of CLP on A549 Cell Apoptosis

As shown in Figure 3, the apoptosis rates of the normal cells were only 5% but it was significantly increased in the CLP-treated groups in a concentration-dependent manner (*P* < 0.05), indicating that CLP induced A549 cell apoptosis. Furthermore, the number of untreated A549 cells at the G1 phase was 67%, which was much lower than those of CLP-treated groups (*P* < 0.05). In other words, CLP obviously caused an accumulation of A549 cells at the G1 phase and decreased in the S phase in a concentration-dependent manner (*P* < 0.05).

### 3.5. Effects of CLP on the Expression of Ras/PI3K/AKT Signals

At 48 h after CLP treatment, the expression levels of Ras, PI3K, AKT, and pAKT were measured by Western blot analysis. In Figure 4, CLP significantly inhibited the expression levels of Ras, PI3K, AKT, and pAKT compared with the control group (*P* < 0.05). However, there were no significant differences of PTEN expression among the control and CLP-treated groups (*P* > 0.05). Therefore, the proapoptotic effect of CLP on lung cancer cells did not depend on the activation of PTEN. Furthermore, after CLP treatment, the expression of Bcl-2, caspase-9, and caspase-3 was significantly reduced but the levels of Bax, clv-caspase 9, and clv-caspase 3 were significantly increased with the increase of CLP concentration (*P* < 0.05).

Since the results of flow cytometry assay showed the cell cycle arrest at the G1 phase induced by CLP, the effect of CLP on the expression of cyclin D1 and CDK4, which were critical for the G1/S transition, was further examined. The results in Figure 4 displayed that the expression of cyclin D1 and CDK4 in the CLP-treated groups was significantly decreased compared with that in the control group (*P* < 0.05), supporting the G1/S arrest of cell cycle exposed by CLP. Notably, the expression of GSK-3*β*, which was related to stabilization of cyclin D1, was significantly upregulated after CLP treatment, indicating that CLP arrested A549 cells at the G1 phase via mediating the GSK-3*β*/cyclin D1/CDK4 pathway.

### 3.6. Antitumor Effects of CLP *In Vivo*

The growth of orthotopic tumor was monitored using the IVIS Lumina LT imaging system. Tumor volumes and weights were represented by radiance. As shown in Figure 5, the tumor growth of the model group was very fast, especially on the 17th day after challenge. As shown in Figure 5, the volumes of tumor in the model group were much higher than the lung. However, both tumor volumes and weights in the CLP-treated groups were much less than those in the model group (*P* < 0.05), indicating that CLP could effectively inhibit tumor growth after 15 days of treatment. Moreover, the tumor volumes and weights in the CLP-H group were significantly decreased compared with those in the DDP group (*P* < 0.05), indicating the stronger potential of CLP on the inhibition of tumor growth in vivo. Interestingly, no significant change was observed in the body weights of tumor-bearing mice between the model and DDP group, while the mice in the CLP-treated group gained more weights than those in the model group (*P* < 0.05). Therefore, CLP would be less toxic to the mice than DDP.

TUNEL staining was used to visualize the cell apoptosis in tumor tissue. As shown in Figure 6, the apoptotic cells (marked as green) hardly existed in the model group, while tumor tissue from the CLP-treated group exhibited a higher percentage of apoptotic cells compared with that from the model group. Therefore, CLP inhibited tumor growth by the augmentation of apoptotic tumor cells.

The tumor cells characterized with markedly large nuclei were aligned tightly and irregularly in the tissues of the model group. However, after CLP treatment, the adhesion of human lung adenocarcinoma cells disappeared and separated from the surrounding cells, the cell volume was reduced, and the nucleoplasm was condensed. In addition, the immunohistochemistry results displayed that the tumor tissues in the CLP-treated groups presented the low brown expression of Ki-67, an antigen indicating the proliferative state of active tumor cells, while those in the tumor tissues of the model group were comparatively high (Figure 7). Similarly, the expressing profiles of pAKT in the tumor tissues were consistent with those of Ki-67. All these results demonstrate that CLP effectively inhibited the growth of A549 cells *in vivo*.

### 3.7. Antibacterial Activity of CLP

In Figure 8, the *α* community richness among the model and CLP-treated groups was considered to assess the effects of CLP on lung dysbiosis in A549 tumor-bearing mice. The levels of 3 indexes (ACE, Chao1, and Shannon), which reflected the microbiota diversities, were significantly increased in the CLP-treated groups as the dose increased compared with those in the model group (*P* < 0.05). The levels of Simpson in CLP-treated groups were decreased compared with those in the model group, but the Simpson levels were significantly different among the CLP-treated groups. Furthermore, the relative abundances of microbes in *Veillonella*, *Streptococcus*, and *Megasphaera* families in the lung tissues of A549 tumor-bearing mice were much higher than those in the CLP-treated mice (*P* < 0.05), while the relative abundances of *Alloprevotella* and *Actinomyces* in the model mice were remarkably lower than those in the CLP-treated mice (*P* < 0.05). Therefore, CLP improved the lung dysbiosis of the mice with lung cancer.

CLP significantly inhibited the growth of *S. pyogenes* and *S. aureus* with MIC values of 1.94 and 2.37 mg/mL and MBC of 1.94 and 4.74 mg/mL. Furthermore, the diameters of bacteriostatic zones of CLP were 12 and 7 mm. These results suggested the potential antibacterial activities of CLP, which would contribute to its regulation on lung dysbiosis induced by cancer cells.

## 4. Discussion

Lung cancer remains the most common malignancies globally. Its molecular mechanisms have been widely studied, and the need for novel therapeutic approaches is also growing. Although platinum- or tyrosine kinase inhibitor-based chemotherapy has been the standard protocol for treating lung cancer, the chemotherapy efficacy is greatly limited by the drug resistance and toxic effects [33–35]. Traditional Chinese medicine combined with chemotherapy has been frequently used to prevent the lung cancer, which could improve the prognosis and decrease the complications of the patients [8]. The efficacy and safety of these adjuvant therapies (such as kanglaite injection, kushen injection, Feiyanning, Javanica oil, and *Astragalus* extract) have been scientifically evaluated [36–38]. Therefore, a therapy should be developed to explore plant-derived compounds with high efficacy, low toxicity, and novelty mechanisms. The herb *C. lanceolata* root contains many bioactive components, including polyphenols, saponins, alkaloids, and polysaccharides [9]. Among these compounds, polyacetylenes were the characteristic and main effective constituents of *Codonopsis* species. Although lobetyolin, a maker polyacetylene glycoside in *C. lanceolata*, reduces hepatic XO activity and inhibits the tumor growth of H22 hepatoma cell xenografts in mice [39, 40], the antitumor activities of *C. lanceolata* and its exact mechanisms have been largely unknown. In the study, for the first time, six compounds (syringin, codonopilodiynoside A, lobetyol, isolariciresinol, lobetyolin, and atractylenolide III) were isolated and identified in the effective fraction of *C. lanceolata* (i.e., CLP). After comparison among the contents and *in vitro* antitumor activities of each compound, lobetyol and lobetyolin contributed approximately 71% to the effects of CLP on lung cancer cell proliferation, indicating that they were the main anticancer compounds in *C. lanceolata*. Then, we investigated the therapeutic potentialities and mechanisms of CLP on A549 cells *in vitro* and *in vivo*. The results showed that CLP obviously suppressed the proliferation, migration, and invasion of A549 cells in the dose- and time-dependent manners. It also inhibited tumor growth in A549 nude mouse xenografts. However, it did not reduce the proliferation of human normal lung epithelial BEAS-2B cells, suggesting its low cytotoxicity.

The proteins involved in the PI3K/AKT pathway are abnormally expressed in human cancers, which participate in every process within cancer cells [41, 42]. PI3K could be activated by Ras and subsequently transduces intracellular signaling by directly binding with the pleckstrin homology domains of various proteins and participates in many physiological processes including cell cycle regulation, DNA repair, cell apoptosis, and glycometabolism [43–45]. AKT inhibits proapoptotic Bcl-2 family members Bax, phosphorylates GSK-3*β*, and negatively regulates caspase-9, which then cleave and activate caspase-3, thereby increasing the expression of antiapoptotic components and cell survival signals [46]. In the study, we found that CLP could not impact the levels of PTEN but could significantly downregulate the levels of Ras, PI3K, and pAKT in A549 cells, indicating that CLP acted as an inhibitor by inactivation of the Ras/PI3K/AKT pathway. Moreover, CLP significantly upregulated levels of Bax, clv-caspase-9, and clv-caspase-3 but downregulated the levels of Bcl-2, caspase-9, and caspase-3 in A549 cells. However, all those profiles could be reversed by PI3K activator 740YP. Therefore, CLP induced the apoptosis of A549 cells by modulating the Ras/PI3K/AKT pathway.

In addition, cell cycle is an essential component involved in the processes of cell proliferation. Uncontrolled cell proliferation is one of the salient features of cancer [47, 48]. Cyclin D1 is an abnormally expressed maker in cancers which promotes the G1 to S phase transition by binding to CDK4 [49]. Photophosphorylation of AKT inhibited the activation of GSK-3*β*, resulting in the stabilization of cyclin D1 [50]. In the study, cell cycle was significantly arrested at the G1 phase in a dose-dependent way after CLP treatment. CLP obviously increased the expression of GSK-3*β* but reduced the levels of cyclin D1 and CDK4 in A549 cells. In addition, in the A549 nude mouse xenograft model, Ki-67 staining results indicated that CLP markedly decreased the proliferative state of cells in tumor tissue sections. Therefore, the antiproliferative effects of CLP would be consistent with the arrest of the G1 phase.

Emerging evidence had showed that lung microbiota plays crucial roles in pathogenesis and progression of lung cancer [51–53]. On one hand, the respiratory bacterial load as well as changes in the bacterial community contributes to tumor cell proliferation, survival, and tissue invasion. Specifically, ACE, Chao1, and Shannon are three common indices reflecting microbiota diversity and richness, while there was a negative correlation between the Simpson level and microbiota diversity. The results showed that CLP treatment could increase the levels of ACE, Chao1, and Shannon but could reduce the Simpson level, indicating that CLP improved lung dysbiosis through increasing microbiota diversity. On other hand, it has been known that the lower airways of patients with lung cancer were enriched with oral pathogenic bacteria *Veillonella*, *Prevotella*, and *Streptococcus* [54–57]. Interestingly, CLP not only decreased the abundance of those oral pathogenic commensals in the lung tissues of tumor-bearing mice but also directly inhibited the growth of *S. pyogenes* and *S aureus*, which are common lung pathogenic bacteria in patients with lung cancer [58, 59], indicating its antimicrobial potential on tumor-related dysbiosis. But its underlying antimicrobial mechanism would be further considered.

In summary, CLP inhibited proliferation and induced apoptosis of A549 cells, which were arrested at the G1/S phase, and suppressed growth of lung cancer in the nude mouse xenograft models. It also significantly upregulated the expression of Bax, GSK-3*β*, clv-caspase-9, and clv-caspase-3 and downregulated the expression of Ras, Pi3K, pAKT, cyclin D1, CDK4, Ras, Bcl-2, caspase-9, and caspase-3 in A549 cells, which all were reversed by the PI3K activator. But CLP hardly altered the expression of PTEN. Thus, it indicated that CLP induced apoptosis of A549 cells via regulating the Ras/PI3K/AKT pathway. Moreover, CLP exerted antibacterial activities in vitro and improved the lung dysbiosis of tumor-bearing mice. It could be a therapeutic candidate for the prevention and treatment of human lung cancer.

## Figures and Tables

**Figure 1:** Effects of CLP on the proliferation of A549 cells. (a) HPLC chromatograph of standards (above) and CLP (below). The peaks marked with 1~6 were syringin, codonopilodiynoside A, lobetyol, (+)-isolariciresinol, lobetyolin, and atractylenolide III, respectively. (b) Effects of CLP on the viability of A549 cells. The A549 cells were treated with 1.25~20 *μ*g/mL of CLP for 24, 48, and 72 h. (c) Effects of CLP on the viability of normal lung epithelial BEAS-2B cells. Cell viability was determined by MTT assay. The BEAS-2B cells were treated with 20 *μ*g/mL of CLP for 24, 48, and 72 h, respectively. (d) Effects of compounds isolated from CLP on viability of A549 cells. The A549 cells were treated with 20 *μ*g/mL of different compounds for 48 h. (e) The contributions of the main bioactivity compounds to the inhibition rates of CLP on the proliferation of A549 cells. The A549 cells were treated with 9.92 *μ*g/mL of syringin, 1.82 *μ*g/mL of lobetyol, and 2.06 *μ*g/mL of lobetyolin for 48 h, which represented their concentrations in 20 *μ*g/mL CLP. (f) The synergistic inhibition of lobetyol and lobetyolin on the proliferation of A549 cells, which was calculated by using CompuSyn software. Data were expressed as means ± SD. The groups marked with different letters suggested significant differences, *P* < 0.05.

**Figure 2:** Effect of CLP on the migration, invasion, and colony formation of A549 cells. (a) Cell migration was determined by a wound healing assay. (b) Cell invasion was determined by a Transwell assay. A549 cells were treated with CLP (2.5, 5, and 10 *μ*g/mL) or DDP (5 *μ*g/mL) for 48 h, respectively. (c) The number of colonies of the A549 cells, which were treated with CLP (2.5, 5, and 10 *μ*g/mL) or DDP (5 *μ*g/mL) for 7 days, was counted under low-magnification light microscope (×100). (d) The quantitative results of migration, invasion, and colony formation assay. Data were expressed as means ± SD. The groups marked with different letters suggested significant differences, *P* < 0.05.

**Figure 3:** CLP induced the apoptosis of A549 cells. (a) The effects of CLP on A549 cell apoptosis. (b) Effect of CLP on cell cycles of A549 cells. Flow cytometry was used to detect apoptotic rates and cell cycles of A549 cells. Data were expressed as means ± SD. The groups marked with different letters suggested significant differences, *P* < 0.05.

**Figure 4:** Effects of CLP on the protein expression of the Ras/PI3K/AKT pathway. (a) Representative bands of key protein expression of the Ras/PI3K/AKT pathway (left). The quantitative results of protein expression in each group (right). (b) PI3K activator 740YP reversed the inhibition of CLP on the protein expression of the Ras/PI3K/AKT pathway (left). The quantitative results of protein expression in each group (right). Data were expressed as means ± SD. The groups marked with different letters suggested significant differences, *P* < 0.05.

**Figure 5:** Antitumor effects of CLP on the A549 tumor-bearing mouse model. The nude mice were randomly divided into five subgroups as follows: model, treated with saline; CLP-L, treated with 10 mg/kg of CLP; CLP-M, treated with 20 mg/kg of CLP; CLP-H, treated with 40 mg/kg of CLP; and DDP, treated with 5 mg/kg of DPP. (a) Tumor growth was monitored every 5 days by using the IVIS Lumina LT imaging system. (b) Tumor growth in the mouse model. (c) Morphological observation of tumor tissue (black arrows). (d) Body weight changes. Data were expressed as means ± SD. The groups marked with different letters suggested significant differences, *P* < 0.05.

**Figure 6:** Effects of CLP on the cell apoptosis of tumor tissues in A549 tumor-bearing mice. TUNEL assay was used to detect apoptotic cells in tumor tissue sections. All images were taken at ×200 magnification.

**Figure 7:** Effects of CLP on cell proliferation in the tumor tissues of A549 tumor-bearing mice. (a) Representative images of HE staining after treatment with CLP. (b) Immunohistochemistry assay was used to detect the proliferative levels of Ki-67 and pAKT in tumor tissue sections. All images were taken at ×200 magnification. (c) Relative expression of Ki-67 and pAKT in tumor tissue sections. Data were expressed as means ± SD. The groups marked with different letters suggested significant differences, *P* < 0.05.

**Figure 8:** Effects of CLP on lung microbiota of A549 tumor-bearing mice. (a) Alpha diversities of lung microbiota. ACE, chao, Shannon, and Simpson indicated the diversities of lung microbiota. (b) Relative abundance of the differently expressed microbiota at the family levels. Data were expressed as means ± SD. The groups marked with different letters suggested significant differences, *P* < 0.05.

## Data Availability

The data is available from the corresponding author upon reasonable request.
